# Sexual Dysfunction in Women with Diabetic Kidney

This article has been retracted.

**DOI:** 10.1155/2014/346834

**Published:** 2014-09-03

**Authors:** Ersilia Satta, Carlo Magno, Alessandro Galì, Antonino Inferrera, Roberta Granese, Carmela Aloisi, Michele Buemi, Guido Bellinghieri, Domenico Santoro

**Affiliations:** ^1^Department of Internal Medicine, Unit of Nephrology and Dialysis, University of Messina, 98100 Messina, Italy; ^2^Dialysis Center, “Dialnefro”, Clinica Mariarosaria, 80045 Pompei, Italy; ^3^Department of Urology, University of Messina, 98100 Messina, Italy; ^4^Department of Pediatric, Gynecological, Microbiological and Biomedical Sciences, University of Messina, 98100 Messina, Italy

## Abstract

Few studies address alteration of sexual function in women with diabetes and chronic kidney disease (CKD). Quality of life surveys suggest that discussion of sexual function and other reproductive issues are of psychosocial assessment and that education on sexual function in the setting of chronic diseases such as diabetes and CKD is widely needed. Pharmacologic therapy with estrogen/progesterone and androgens along with glycemic control, correction of anemia, ensuring adequate dialysis delivery, and treatment of underlying depression are important. Changes in lifestyle such as smoking cessation, strength training, and aerobic exercises may decrease depression, enhance body image, and have positive impacts on sexuality. Many hormonal abnormalities which occur in women with diabetes and CKD who suffer from chronic anovulation and lack of progesterone secretion may be treated with oral progesterone at the end of each menstrual cycle to restore menstrual cycles. Hypoactive sexual desire disorder (HSDD) is the most common sexual problem reported by women with diabetes and CKD. Sexual function can be assessed in women, using the 9-item Female Sexual Function Index, questionnaire, or 19 items. It is important for nephrologists and physicians to incorporate assessment of sexual function into the routine evaluation protocols.

## 1. Introduction

The prevalence and incidence of diabetes is rather similar in the two sexes [1]. However, the long-term impact of diabetes on complication is more gender specific. Men in comparison with women seem to be at higher risk for microvascular complications, such as nephropathy [2], severe retinopathy [3], and sexual dysfunction [4]. Diabetic nephropathy is a major complication of diabetes mellitus (DM), affecting about 15%–25% of type 1 and 30%–40% of type 2 diabetic patients, and diabetic nephropathy accounts for approximately 44% of all cases of end stage renal disease (ESRD) [5]. Disturbances in sexual function are associated frequently with diabetic nephropathy and CKD [6]. Male patients with diabetic nephropathy and CKD suffer from reduced libido, erectile dysfunction, and difficulty reaching the orgasm. In females with diabetic kidney, dyspareunia, amenorrhea, reduction of libido, and a delay in sexual development are frequently observed. Sexual function of women with diabetes, however, has received less attention in clinical studies. Moreover results are less conclusive than studies in men, likely due to several factors, including a lack of standardized definitions of female sexual dysfunction, absence of well-validates scales, and social taboos regarding female sexuality [7].

## 2. Female Sexual Dysfunction

Female sexual dysfunction (FSD) has been described in diabetic women since the early 1980s. Sexual disorders reported in women with diabetes include the reduction or loss of sexual interest or desire, arousal or lubrication difficulties, dyspareunia, and loss of the ability to reach orgasm [7].

FSD is defined as a disorder of sexual desire, arousal, orgasm, and/or sexual a pain. In 2010, the Third International Consensus of Sexual Medicine accepted revised definitions of FSD, emphasizing a model based on a circular pattern of the sexual female response, in which different phases of sexual function can overlap. More recently, the* Diagnostic and Statistical Manual of Mental Disorders, Fifth Edition *(DSM-5), released newer and revised definitions, in which sexual desire and arousal disorders have been combined into the “female sexual interest/arousal disorder” category, and vaginismus and dyspareunia have been grouped into the “genitopelvic pain/penetration disorder” category. Moreover, all of the sexual dysfunctions outlined in the DSM-5 require a minimum duration of approximately 6 months, and more precise severity criteria must be met in order to provide useful thresholds for making a diagnosis and for distinguishing transient sexual difficulties from more persistent sexual dysfunction [8, 9].

FSD has been associated with both type 1 and type 2 diabetes. A recent meta-analysis that included 26 studies, 3,168 diabetic women, and 2,823 controls showed that FSD is more frequent and is associated with a lower Female Sexual Function Index (FSFI) score in diabetic women than in controls. In particular, the risk for FSD was 2.27 (95% confidence interval (CI): 1.23–4.16) and 2.49 (95% CI: 1.55–3.99) in type 1 and type 2 diabetic women, respectively. Furthermore, the risk for FSD was 2.02 (CI: 1.49–2.72) when considering “any diabetes” (which represented the two forms of diabetes together). Interestingly, an increased risk of FSD was found in premenopausal women with “any diabetes,” but not in postmenopausal women. Moreover, at the statistical analysis among the independent variables, only BMI was significantly associated with the FSFI effect size (*P* = 0.005), suggesting that the higher frequency of FSD and lower FSFI score found in diabetic women may be related to body weight. Several studies have already shown an increased prevalence of FSD in women affected by obesity and metabolic syndrome [10]. Studies that have focused on type 1 diabetic women provided a valid opportunity to investigate the role of diabetes on sexual function, independent of other associated comorbidities. In type 1 diabetic women, FSD appears to be correlated mainly psychological factors, such as depression, anxiety, and marital status [11]. Results from a large prospective study of 625 women with type 1 diabetes showed that depression was the major predictor of sexual dysfunction [11].

## 3. Pathophysiology

Pathogenesis of FSD is related to decreased libido, low arousability, decreased vaginal lubrification, orgasmic dysfunction, and dyspareunia. The causes implicated in such disturbances are peripheral neurological disease, vascular impairment, and psychological complaints.

Several studies showed that circulating concentration of estradiol are decreased in women with type 1 DM, suggesting that diabetes may be associated with dysregulation of sex hormone biosynthesis [12]. Similar observations were made in patients with CKD and type 1 DM. Women with diabetes type 1 have impaired ovarian function, delayed age at menarche, more risk of menstrual irregularities, and complication in pregnancy such as spontaneous abortion, stillbirths, and congenital anomalies, when age matched with nondiabetic women. A set of validated instruments including the Female Sexual Distress Scale (FSDS) and Beck's Inventory for Depression (BDI) were used as basic methods. During the follicular phase, patients and control subjects had similar FSFI scores. During the luteal phase, patients had significantly lower FSFI scores and significantly higher FSDS scores, while BDI was equal. During the follicular phase, patients had lower estrogenic profile, as well as delta4-androstenedione, DHEAS, and fT4 and fT3 than control subjects. During the luteal phase, total testosterone levels were higher in patients than control subjects, while 17-Beta estradiol and progesterone levels were lower in patients than in control subjects [13].

The endocrinological basis of FSD in diabetic disease was mostly investigated in the study conducted by Salonia et al. [13]. Sexual function and endocrine profile in women with type 1 diabetes were studied during follicular and luteal phases of menstrual cycle and compared to control group.

In women with diabetic nephropathy and CKD, decrease of libido, amenorrhea, disturbances in menstruation, and fertility are caused by elevated levels of follicle-stimulating hormone (FSH) and luteinizing hormone (LH). Midcycle LH surge cannot be mitigated with endogenous administration of estrogen, confirming a central hypothalamic derangement. The major menstrual abnormality in diabetes and CKD is anovulation, with consequence of infertility. Clinical manifestations of sexual dysfunction in women include premature menopause, skin wrinkling, urinary incontinence, hot flushes, sleep and cognitive disorders, and cardiovascular disease [12]. The reduction of libido is frequently observed, while the pregnancy is rare (spontaneous abortion is a common eventuality). Few studies carefully examined ovarian function in women with diabetic nephropathy; this lack of data reflects probably the complexity of studying the reproductive system in women. Both the smooth muscle relaxation of female genitalia erectile tissue and the enhancement of genital blood flow are dependent upon the action of nonadrenergic/noncholinergic neurotransmitters, such as vasoactive intestinal polypeptide b (VIP) and nitric oxide (NO). The regulation of blood flow and clitoral erectile function is governed by the same NO/cyclic guanosine monophosphate (cGMP) pathway in women as well as that involved in erectile function in men. NO and phosphodiesterase type 5 (PDE5) have been identified in human clitoral smooth muscle, indicating a key role of NO in female sexual function [14]. Normal levels of various hormones are also required for physiologic sexual activity. Diabetes and CKD may affect all of these integrated systems, leading to sexual dysfunction. The mechanisms involved include hyperglycemia, infections, vascular and neurological damage, and hormonal disorders [15].

## 4. Sex Hormones in the Diabetic kidney

Several studies focused on the association between sex hormones and diabetic renal disease. First, puberty is the turning point for the development of diabetic nephropathy. Second, the protection of the female sex against the development of renal disease is missing in setting of diabetes [16]. Third, CKD, secondary to diabetes, is associated with sexual dysfunction and altered sex hormone profiles. Despite the fact that it is unclear whether diabetic nephropathy is characterized by an imbalance in sex hormone levels and whether restoring this imbalance may be renoprotective, few studies tested the effects of estrogens in diabetic nephropathy [6, 17]. Short-term administration of estrogens in recombination with a synthetic progestin has been shown to reduce proteinuria and improved creatinine clearance in postmenopausal women with type 2 diabetes. Similarly, the Insulin Resistance Atherosclerosis Estradiol exerts its actions through both Er alfa and Er beta receptors, which are predominants in the kidney of female rats, whereas only Er beta receptors are predominants in male [16]. Not all studies, however, support the beneficial effects of estrogens in the diabetic kidney.

The use of oral contraceptives, containing high doses of estrogen, has been linked to the development of macroalbuminuria [16].

Ovarian failure in women with diabetic kidney and CKD can be associated with abnormalities at several sites in the hypothalamic-pituitary-ovarian axis.

During the follicular phase of the ovarian cycle, baseline plasma levels of estradiol, progesterone estradiol, and FSH are comparable between premenopausal women with diabetic disease. During the midcycle LH surge, however, the LH levels of premenopausal women with diabetes and CKD are far below those of normal women. After administration of clomifene, which can be used to evaluate the responsiveness of the hypothalamic-pituitary axis, plasma levels of LH and FSH increase significantly in patients, which indicates that the negative-feedback effect of estrogen on the hypothalamus is intact. Secretion of gonadotropin-releasing hormone (GNRH) has both tonic and cyclic components. The tonic component regulates basal gonadotropin secretion and is controlled by negative estradiol feedback mechanism. The cyclic component is dependent on estrogen secretion; the increase in estrogen levels in the middle of the menstrual cycle is responsible for enhanced secretion of GNRH and subsequent LH surge [6, 17].

After an estrogen stimulation test, normal individuals experience a surge in plasma LH levels; by contrast, plasma LH levels do not rise and plasma FSH levels are suppressed after administration of estrogen to women with diabetic nephropathy. The absence of an increase in LH levels in these patients strongly indicates a defect in the positive hypothalamic feedback mechanism.

High levels of serum prolactin, present in 80% of women with diabetes and CKD, might contribute to ovulatory dysfunction and decreased libido in this population.

## 5. Psychological Factors

Psychological factors can have a substantial effect on the sexual function in patients with diabetes and CKD. It has been noted in several studies that 20–30% of patients with diabetes and CKD suffer from clinical depression. Psychometric profile includes mood deflection, major depression, interpersonal issue and psychological aspect of living with diabetes and CKD [17].

Two major studies by Enzlin et al. [11] showed that women with DM1 either with or without SD reported more depressive symptoms than men with and without SD, respectively.

Enzlin et al. [11] reported a significantly higher incidence of depressive symptoms in women with DM1 who had sexual problem than in women without sexual dysfunction [11]. However, depression is a well-known determinant of decreased desire impaired arousability in women with diabetes. Salonia et al. suggest, according to the Female Sexual Distress Scale (a 12-item instrument to measure sexually related personal distress in women, that sexual distress is similar between patients and control subjects during the follicular phase. In women with DM1 sexual distress correlated significantly with a reduction in libido scores (*r* = −0.44, *P* = 0.034) and lower lubrification scores (*r* = 0.45, *P* = 0.032).

Associations were found between FSD and a variety of other quality of life parameters, such as mental and physical components of the 36-item short-form (SF-36) health survey and depression scores.

Depression is strongly associated with diabetes. Most epidemiological studies showed that psychosocial factors are the main contributors to sexual dysfunctions in both type 1 and type 2 diabetes. Depression seems to be the main determinant of sexual dysfunction in women with diabetes. Diabetic complications may also affect health and relationship status, quality of life, and a woman's self-image, generating a vicious cycle that may have detrimental effects on sexual performance.

## 6. Diagnosis and Evaluation of Sexual Dysfunction

The first step in the evaluation of sexual dysfunction in patients with diabetes and CKD is to obtain a detailed sexual history about the sexual desire, arousal and orgasmic capabilities, and fertility. Changes in the frequency of intercourse need to be determined. Often the patients are very reluctant to tell such concerns. The physicians should determine the time of the onset of these problems in relation to the stage of disease [17–19]. The domains of sexual function in women include desire, arousal, pain, and satisfaction. These can be assessed using the 9-item FSFI. There are several validated screening tools that focus on HSDD, which is the most common sexual concern of women of all ages (Table 1) [20–22].

In addition, the medical history should focus on the patient's past and present medical illness, that is, chronic/medical illness, such as anemia; neurological illness or lumbosacral disc disease; endocrinological disease, like hypogonadism, hyperprolactinemia, and thyroid disorders; atherosclerotic vascular risk, hypercholesterolemia, hypertension, hyperhomocysteinemia, smoking habits, or family history. Current drug therapy should also be reviewed in detail. Drugs such as cimetidine, tricyclic antidepressant, phenothiazines, and metoclopramide are often implicated in SD in female.

Finally, it is important to investigate patients for presence of psychosocial problems (depression, psychiatric illness) and current stressors factor (loss of job or home and so on).

## 7. Management of Sexual Dysfunction in Women

Few studies address decreased libido and sexual function in women with diabetic nephropathy and CKD. Surveys on “quality of life” suggest that discussion of sexual function and other reproductive issues are key components of psychosocial assessment and that education on sexual function in the setting of diabetic nephropathy and CKD is widely needed [23]. Pharmacologic therapy with estrogen/progesterone and androgens along with correction of anemia, ensuring adequate dialysis delivery, and treatment of underlying depression are important. Changes in lifestyle such as smoking cessation, strength training, and aerobic exercises may decrease depression, enhance body image, and have positive impacts on sexuality [24, 25]. Women with diabetic nephropathy who suffer from chronic anovulation and lack of progesterone secretion may be treated with oral progesterone at the end of each menstrual cycle to restore menstrual cycles. It is not clear whether unopposed estrogen stimulation of the endometrium (due to anovulatory cycles) predisposes women with diabetic nephropathy to endometrial hyperplasia or endometrial cancer. Routine gynecologic follow-up is recommended in these cases, and some women may also benefit from the use of a progestational agent several times a year to mitigate the effects of estrogen on the endometrium [23–28].

Low estradiol levels in amenorrhoeic women on diabetes leads to vaginal atrophy and dyspareunia. Topical estrogen cream and vaginal lubricants may be helpful in this situation. Women with diabetic nephropathy who do have menstrual cycles should be encouraged to use contraception; because of poor pregnancy outcomes, restoring fertility is not an advisable therapeutic goal. HSDD is the most common sexual problem reported by women with diabetes and CKD. Testosterone replacement therapy to treat HSDD has been effective in some women without diabetes and CKD [29]. However, long-term safety data on the use of androgens in women with diabetes and CKD are very limited (Table 2).

## 8. Conclusions

FSD pathogenesis in diabetes is complex, and current studies have not yet clarified all of the pathological pathways involved; these studies are limited by the small sample sizes, lack of standardized definitions of sexual dysfunction, and inadequate characterization of diabetes, especially regarding glycemic control, the presence of complications, and the presence of depression. In contrast to what is described in men, female sexual function appears to be more related to social and psychological components than to the physiological consequence of diabetes. In conclusion, psychological concerns may play a significant role in the development of FSD in both type 1 and type 2 diabetes. This is in line with the complex nature of female sexuality, which is largely dependent on psychological and cultural factors, even more so than male sexuality.

## Figures and Tables

**Table 1:** Screening tools for FSD.

(i) Decreased Sexual Desire Screener (DSDS): 5 questions, self-administered, assesses for generalized acquired HSDD [29].	
(ii) Female Sexual Function Index (FSFI): 19 questions, self-administered, assesses all of the dimensions of female sexual function including sexual satisfaction [20].	
(iii) Sexual Interest and Desire Inventory-Female (SIDI-F): 13 items, clinician administered, assesses severity of female HSDD [21].	
(iv) Brief Hypoactive Sexual Desire Disorder Screener: 4 questions, self-administered HSDD in postmenopausal women [21].	
(v) Brief Profile of Female Sexual Function (B-PFSF): 7 questions, self-administered HSDD in postmenopausal women [21].	
(vi) Female Sexual Distress Scale-Revised (FSDS-R): 13 questions, self-administered, assesses distress associated with female SD [19, 21, 22, 26, 30].	

**Table 2:** What the guidelines say you should do: treatment of sexual dysfunction in women and the opportunity for psychosexual and/or couples counseling.

(i) The generalized use of testosterone by women has been advised against, because of inadequate indications and lack of long-term data. However, postmenopausal women who are distressed by their decreased sexual desire and who have other identifiable causes may be candidates for testosterone therapy. Androgens which may also be used by those women are hypogonadal as a result of pituitary problems in premenopause.	
(ii) Although there is no consistent correlation between sexual functioning and levels of androgens (free and total testosterone, androstenedione, dehydroepiandrosterone, and SHBG) across wide age range, in some women androgen therapy can improve sexual desire.	
(iii) Transdermal patches and topical gel or creams are preferred over oral products because of first pass hepatic effects documented with oral formulation.	
(iv) The major side effects of androgens are hirsutism and acne. No safety with regard to testosterone implants. There is no indication for increased frequency of breast cancer [20, 21, 27–29].	
